The article "Fibroblasts in Scar Formation: Biology and Clinical Translation" was retracted in 2023. Reasons: suspected computer-generated content; unreliable results or conclusions; concerns about the data; concerns about the results or conclusions.

# Fibroblasts in Scar Formation: Biology and Clinical Translation

**DOI:** 10.1155/2022/4586569

**Published:** 2022-05-12

**Authors:** Huan Qian, Yihan Shan, Ruicheng Gong, Danfeng Lin, Mengwen Zhang, Chen Wang, Lu Wang

**Affiliations:** ^1^Department of Plastic Surgery, The Second Affiliated Hospital, School of Medicine, Zhejiang University, Hangzhou, China; ^2^Wenzhou Medical University, Wenzhou, China; ^3^Starbody plastic surgery Clinic, Hangzhou, China; ^4^Department of Breast Surgery, The First Affifiliated Hospital of Wenzhou Medical University, Wenzhou, China

## Abstract

Scarring, which develops due to fibroblast activation and excessive extracellular matrix deposition, can cause physical, psychological, and cosmetic problems. Fibroblasts are the main type of connective tissue cells and play important roles in wound healing. However, the underlying mechanisms of fibroblast in reaching scarless wound healing require more exploration. Herein, we systematically reviewed how fibroblasts behave in response to skin injuries, as well as their functions in regeneration and scar formation. Several biocompatible materials, including hydrogels and nanoparticles, were also suggested. Moreover, factors that concern transformation from fibroblasts into cancer-associated fibroblasts are mentioned due to a tight association between scar formation and primary skin cancers. These findings will help us better understand skin fibrotic pathogenesis, as well as provide potential targets for scarless wound healing therapies.

## 1. Introduction

Many situations can cause skin injuries, and most human skin wounds heal with the process of scarring. While some scars reach complete regeneration, many others undergo pathological tissue repairs, which occur with hypertrophic and keloid scars [1]. Treatment often involves surgical resection, laser therapy, radiation therapy, physical therapy (i.e., pressure therapy), and medication (i.e., triamcinolone injections) [2–5]. Currently, a number of animal studies have reported the molecular basis of scar-free healing [6–9]. Several factors, including growth factors, cytokines, cells (especially fibroblasts), and the extracellular matrix (ECM), contribute to scar formation. However, any preventive and therapeutic strategies to date remain unsatisfactory [10], which brings significant challenges to clinical practice. Additionally, differentiation towards cancer-associated fibroblasts (CAFs) may have an adverse function in skin healing. Yet, given the rapid development of nanotechnology, the use of nanodrugs may facilitate scar-free wound healing [11, 12].

## 2. Fibroblasts in Wound Healing and Pathological Scar Repair

### 2.1. Wound Healing Process

The wound healing proceeds across three partially overlapping phases, including inflammation, re-epithelialization, and tissue remodeling [13]. It is considered to be a rather complex, but well-organized physiological process that involves mediators, ECM components, growth factors, and proteinases [12, 14].

The inflammation often occurs within 48 h after injury and is characterized by a hypoxic and ischemic environment [15]. A fibrin clot is formed, and platelets are able to be activated by release of several growth factors, including transforming growth factor (TGF-*α* and TGF-*β*), epidermal growth factor (EGF), platelet-derived growth factor (PDGF), and fibroblast growth factor (FGF) [16–18]. Neutrophils and macrophages are also activated and summoned to curb the infection [19]. The re-epithelialization stage is characterized by the formation of new tissues. The early event involved the migration of keratinocytes to cover the skin surface [20]. Under stimulation of PDGF and FGF from previously attracted inflammatory cells, granulation tissue is gradually formed by involvement of angiogenesis, as well as migration of fibroblasts [21]. With the accumulation, differentiation, and proliferation of fibroblasts, new ECM is produced, and wounds become slowly contracted [22]. The remodeling phase can last for a year or even longer, and apoptosis develops in most endothelial cells, macrophages, and fibroblasts, at this stage [23]. The collagen III in the newly synthesized ECM is gradually replaced by more robust collagen I, which enhances tensile strength of the healed skin [24].

### 2.2. Fibroblasts in Wound Healing

Fibroblasts, which are known as connective-tissue-resident cells that generate ECM the scaffolding of the body, play important roles in wound healing [25]. The normal dermis can be divided into three layers containing different fibroblasts, including the papillary dermis (with papillary fibroblasts), reticular dermis (with reticular fibroblasts), and hypodermis/white adipose layer (with preadipocytes and adipocytes) [26, 27]. The histological structure of skin scars can be quite distinguishable. Numerous active fibroblasts and lymphocytes are located within the superficial dermis, while the middle layer contains abundant fibroblasts and ECM. Only a few dermal cells lie within the deep layer [28]. After injuries, the reticular fibroblasts gather and produce ECM [26, 29]. By expressing *α*-smooth muscle actin (*α*-SMA) and large amounts of ECM proteins, dermal regeneration is initiated. This phenomenon was observed by Driskell et al. and Emanuel et al. [27, 30]. The papillary fibroblasts are then recruited in the subsequent re-epithelialization phase [27]. Goss et al. suggested that, unlike reticular fibroblasts, papillary lineage-derived fibroblasts significantly enhance the regeneration of blood vessel-associated pericytes, which indicates a higher angiogenic potential during the second phase of wound healing. This result is also supported by Emanuel et al. [31, 32]. Additionally, modulation of developmental pathways, including canonical wingless-related integration site (Wnt) transcription factor lymphoid enhancer factor 1 (Lef1) in papillary fibroblasts, enables better skin repair [33].

The resident fibroblasts can also facilitate skin repair by wound contraction and crosstalk with immune cells by differentiating themselves into myofibroblasts, which are the major force in scarring [34, 35]. As they are a distinct subpopulation of myofibroblasts, adipocyte precursors have been proven to contribute to wound repair and ECM production and regulation [35, 36]. Maksim et al. have also indicated that new hair follicles in a wound can reprogram the myofibroblasts into adipocyte differentiation by activating the bone morphogenetic protein signaling pathway [37].

Besides the afore-mentioned fibroblasts, other types of fibroblasts have also been reported to affect skin repair. For example, fascia fibroblasts help scarring by swarming to the skin surface in the case of deep wounds [38]. Among chronic open wounds, however, Engrailed-1 (En1-)-positive fibroblasts were detected both in the skin, as well as in the underneath fascia, which can help prevent fascia fibroblasts from migrating upwards, thus inhibiting wound repair [38].

### 2.3. Fibroblasts in Pathological Scar Repair

Pathological scar formation (i.e., hypertrophic scarring or keloids) may develop as long-term sequelae of delayed wound healing [39]. It is mainly featured by excessive proliferation of fibroblasts, as well as massive deposition of ECM (mostly collagen), reduced tensile strength and elasticity, and a lack of hair follicles [40].

Fibroblasts are heterogeneous cells, whether by cell lineage or by molecular phenotype [25]. For example, fibroblasts that are derived from embryonic precursors that express En1 have been reported to be the culprit in skin fibrosis, and targeted suppression/inhibition can effectively reduce formation of scars during wound healing [41]. Leavitt et al. demonstrated the inherent fibrotic characteristics of paired-related homeobox-1 (Prrx1-)-expressing fibroblasts during wound repair by lineage tracing and single-cell transcriptomics technology [42]. Deeper understanding of skin fibroblast lineages may help provide increased clues with regard to regenerative therapies that target subpopulations [43].

Surface markers are often frequently utilized to further identify and isolate fibroblast populations. For example, the upper (papillary) and lower (reticular) dermis can be subdivided by differentially expressed markers [27]. As is confirmed by lineage tracing, the papillary fibroblasts are characterized by an a8 integrin subunit, dipeptidyl peptidase 4 (Dpp4), Lrig1, and B lymphocyte-induced maturation protein 1 (Blimp1), while Dlk1 and Sca1 are selective markers for the lower dermis [27, 29, 44]. Functional analysis and expression profiling studies have suggested that FAP+CD90- cells represent a population of papillary fibroblasts that display proliferative potential. On the other hand, FAP-CD90+ fibroblasts from the reticular lineage may undergo adipogenic differentiation [45].

Myofibroblasts, the primary effector cells in scar formation, mainly derive from fibroblasts with distinct markers and functions. According to a study led by Shook et al., the most abundant populations include adipose precursors (Aps) that express CD26, as well as cells with highly expressed CD29 on the surface (CD29-High) in the wound bed [35]. The significant upregulation of Connexin 43 (Cx43) in specialized fascia fibroblasts are known to be responsible for scar formation, while inhibition of Cx43 prevents collective migration of fascia En1-positive fibroblasts, which disrupts the repair of deep injuries [46]. Other wound-associated biomarkers include SMA*α*+, FAP+, and FSP1+ [22]. Meanwhile, high expression of FOXF2 is measured in scar fibroblasts, and knockdown of FOXF2 demonstrates declined scars and reduced collagen I. In contrast to normal skin, abnormal scars fail to drop the immature scar phenotype, which is characterized by a CD34 and *α*-SMA dermal region [47].

## 3. Regulation of Fibroblasts in Wound Healing and Scar Formation

### 3.1. Microenvironment

The microenvironment in the wound area often regulates behaviors of fibroblasts through the use of mechanical forces, interaction with other cells (i.e., keratinocytes), and numerous substances, including cytokines. Mechanical forces are able to cause scarring via myofibroblast differentiation and collagen overproduction. The shift of fibroblasts towards profibrotic phenotypes is driven by ERK-YAP activation in human cells [48]. Consisting of more than 80% of epithelial cells, keratinocytes make a great contribution to not only skin protection, but also to re-epithelialization and wound closure after injuries [49]. The secretion of the high-mobility group box chromosomal protein 1 (HMGB1) by keratinocytes is known to trigger an *α*-smooth muscle actin promoter by motivating fibroblasts by promoting the nuclear import of MRTF-A, as well as increasing nuclear accumulation of MRTF-A/SRF complexes [50]. Interestingly, thinner skin and reduced collagen density were found among mice with focal adhesion kinase (FAK)-deleted keratinocytes, which actively participate in mechano-transduction and ECM production [51, 52].

In addition, cytokines and cell adhesion molecules are also reported to play roles in ECM deposition, fibroblast differentiation, and cell migration. TGF-*β*-induced release of IL-11 is significantly upregulated in hypertrophic scars, which activates the enrichment of CD39+ fibroblasts within the upper dermis and secretes a large amount of ECM [53]. CD44 is a cell surface adhesion receptor that has been implicated in leukocyte recruitment, T cell extravasation, and hyaluronic acid metabolism. Mice that lack CD44 exhibit reduced collagen degradation, which leads to increased accumulation during and after wound closure [54]. CXCL4 has been validated to stimulate endothelial-to-mesenchymal transition in fibrotic tissues. Myofibroblast differentiation and collagen synthesis are directly induced, indicating that CXCL4 may be a potential therapeutic target for the treatment of fibrosis and scars [55]. Meanwhile, N-cadherin has been shown to be critical in injury-triggered swarming, as well as migration of fascia fibroblasts that progressively contract the skin and form scars [56].

### 3.2. Signaling Pathway

Key aspects of fibroblast biology, which consists of cell differentiation, migration, proliferation, and ECM secretion, are regulated by several signaling pathways during wound healing and scar formation. In general, aggravated scarring is thought to be associated with c-Jun N-terminal kinase (JNK), TGF-*β*, Wnt, and Hippo pathways (with enhanced fibroblast migration, increased transition into myofibroblasts, and ECM rearrangement), whereas JUN is related to better repair. Contractile myofibroblast state transition is needed for fibroblasts to fully function, while the aberrant and sustained switch contributes to both scarring, as well as the development of certain cancers.

As previously reported, differentiation is dominantly controlled by the TGF-*β* pathway. TGF-*β* pathway controls a wide variety of cellular processes, ranging from cell proliferation and differentiation to tissue homeostasis and regeneration via SMAD-dependent (canonical) and independent (noncanonical) signaling [57, 58]. Based on functional analysis, boosted myofibroblast differentiation and excessive deposition of ECM have been observed due to increased levels of TGF-*β*1, mediated by Dpp4 and urokinase (PLAU) *in vitro* [59].

Relative therapeutic strategies include targeted inhibition of TGF-*β* at the genetic and cellular levels. As a TGF-*β* profibrotic signaling-related microRNA, MiR-125b is known to be required for fibroblast-to-myofibroblast transition [60]. The suppression of miR-1224-5p is indicated to decrease proliferation, as well as invasion of keloid fibroblasts, by inhibiting the TGF-*β*1/Smad3-related pathways, thereby further emphasizing the importance of miRNAs as the potential target [61]. Similar activation of the myofibroblast transition has been suggested in other signaling pathways. For example, scars can develop when the translocation of *β*-catenin in fibroblasts is enhanced by Wnt, thereby leading to proliferation, migration, and transition of fibroblasts into myofibroblasts, as well as deposition of type I collagen [62]. Reduced expression of collagen I and III was observed in a biomimetic nanodrug delivery system with increased efficacy on hypertrophic scars by regulating Wnt/*β*-catenin and JAK2/STAT3 pathways [63]. Interestingly, Sun et al. recently discovered that activation of sonic hedgehog can eliminate the negative effect brought by long-term Wnt signaling [64]. In another study, David et al. demonstrate that induced fibroblast activation and upregulated expression of myofibroblast marker proteins are present in samples that are treated with extracellular signal regulated kinase (ERK) or JNK inhibitors and that treatment with a p38 inhibitor can sufficiently inhibit fibroblast activation [65]. It is also worth mentioning that the activation of fibroblasts differentiation mediated by ERK or JNK inhibition can be partially antagonized by cotreatment with a small molecule inhibitor of TGF-*β*R1, indicating that there is underlying crosstalk between these various signaling pathways [66]. In the meantime, stimulation on other fibroblast subpopulations is also proposed. Hippo signaling pathway has emerged as being central to regeneration, in which an elevated nuclear level of YAP and TAZ has been observed [67]. On the other hand, YAP inhibition blocks activation of En1 and promotes ENF-mediated repair, which induces recovery of normal dermal ultrastructure [68]. Additionally, administration with the nuclear Yap-TEAD inhibitor verteporfin prolonged myofibroblast persistence and converted tissue regeneration to fibrosis *in vivo* [69]. JUN initiates hypertrophic scar formation by regulating CD36, modulating distinct fibroblast subpopulations, boosting reticular fibroblasts, and decreasing levels of lipofibroblasts [70].

Given the role of fibroblasts and signaling pathways, any abnormalities that concern fibroblasts (dysregulation of gene expression, altered differentiation, adverse microenvironment, and deflected signaling pathways) can affect regeneration and even cause pathological scarring. For instance, both *in vivo* and *in vitro* experiments conducted by Schulz et al. indicated that a lack of *α*11*β*1 related to defective TGF-*β*-dependent JNK signaling prevents effective conversion from dermal fibroblasts to myofibroblasts, causing poor collagen remodeling [71]. In another study, fibroblasts with conjugation-deficient ISG15 were associated with increased reactive oxygen species (ROS) levels and fewer ROS scavengers, which manifested as ulcerating skin lesions [72]. It has also been shown that selective loss of fibroblasts from the upper dermis after acute and chronic ultraviolet radiation can cause skin injury [73].

## 4. Fibroblasts and Cancer-Associated Fibroblasts

Despite the mechanisms that are involved in regeneration and scar formation, the dysfunction of fibroblasts can lead to a worse case——cancer. It is known that the process of wound healing (scarring in particular) and cancer progression shares several common characteristics, including promoting proliferation and migration of epithelial cells and activation of fibroblasts and excessive ECM deposition, angiogenesis, and lymphangiogenesis, as well as increase in levels of various types of immune cells [74, 75]. From this phenomenon, we can draw the hypothesis that cancers and scarring may share some similar mechanisms.

The microenvironment plays a significant role in both wound healing and tumorigenesis through intracellular communication. The past decade has witnessed a soaring interest in studies that concern the tumor microenvironment and CAFs, a major component and the main cell type that produces ECM. CAFs derive from a diverse group of cells (mainly intrinsic fibroblasts and stellate cells) under either endogenous or exogenous stimulation. Although some biomarkers of CAFs, such as fibroblast activation protein (FAP), *α*-SMA, fibroblast specific protein 1 (FSP1), and platelet-derived growth factor receptor (PDGFR), have been proposed, the complex heterogeneity has not yet been fully revealed [76].

Recent studies demonstrate the process and effect of reprogramming of skin fibroblasts into CAFs [77, 78]. A notable example is the strong upregulation of tumor necrosis factor (TNF)-receptor associated factor 6 (TRAF6) in CAFs in melanoma, which enhances proliferation and migration of fibroblasts, and is accompanied by increased expression of matrix metalloproteinase and *α*-SMA. Furthermore, FGF19 has been shown to be a key cytokine regulated by TRAF6 through NF-*κ*B [79]. Twist1, another key regulator of CAFs, can directly upregulate Prrx1 expression, and subsequently enhance expression of Tenascin-C (TNC), which, in turn, increases the expression of Twist1. Thus, a Twist1-Prrx1-TNC positive feedback loop (PFL) is developed, which leads to the sustained activation of fibroblasts, and the transformation into CAFs [80]. Notch1 is capable of blocking DNA damage response and ensures growth arrest by suppression of ATM-FOXO3a association and the downstream signaling cascade. The amplification of Notch1 is observed in CAFs from squamous cell carcinomas, as well as normal dermal fibroblasts (to a lesser extent), and exposure to UVA (ultraviolet A) expands the effect in normal dermal fibroblasts, while the squamous cell carcinomas appear to be resistant [81]. Activin A is overexpressed in different skin cancers, including basal cell carcinomas, squamous cell carcinomas [82], and melanoma [83–85]. It has been reported to reprogram fibroblasts into protumorigenic CAFs via a Smad2-mediated transcriptional regulation of the formin mDia2, promoting filopodia formation and cell migration. Blockade of this paracrine activin A-mDia2 axis suppresses cancer cell malignancy and squamous carcinogenesis *in vitro* and *in vivo* [86, 87]. As for facilitated invasiveness, keloid tissue-derived fibroblasts (KF) with upregulated LARP6 expression demonstrates enhanced cell proliferation and invasive behavior in cell culture system, while knockdown of LARP reverses this effect, with reduced deposition of type I collagen and inhibition of proliferation and invasion ability [88]. In another study, Tan et al. revealed the role of PPAR*β*/*δ* in the epithelial-mesenchymal communication involved in cellular redox homeostasis. Mice with PPAR*β*/*δ*-deleted fibroblasts indicated retarded growth of tumors [89]. Decreased melanoma invasion is detected, with an upregulation of collagen-cleaving MMP1 expression and subsequent degradation of local collagen (COL1A1) due to damaged dermal fibroblasts by UVR [90].

On the other hand, substances that enhance the genomic stability are likely to prevent CAF transformation. E3 ubiquitin ligase Smurf2 protects human dermal fibroblasts (HDFs) from malignant transformation by regulating E3 ubiquitin ligase RNF20 and histone methyltransferase EZH2, thereby stabilizing chromatin. Depletion of Smurf2 converts HDFs into a tumorigenic entity [91]. Down-modulation of CSL/RBP-J*κ*, the effector of canonical NOTCH signaling, with intrinsic transcription repressive function, harms genomic stability and causes conversion of dermal fibroblasts into CAFs [92]. A deficiency of CLEC2A, the ligand of activating NK cell receptor NKp65, may participate in the fibroblast reprogramming process. The expression of CLEC2A on fibroblasts may be downregulated by TNF-*α*, IL-1*α*, and IL-1*β*, but not by TGF-*β in vitro*. It has been suggested that CLEC2A can accelerate the engulfment of cancer cells by NK cells at early tumorigenesis stages, at which time fibroblasts do not change to the CAF phenotype [93].

## 5. Materials in Scarless Wound Healing

As mentioned above, wound repair is an extremely well-organized process that is mainly conducted by fibroblasts, and scars are the result of dysregulation with excessive ECM deposition and fibroblast proliferation. The primary goal of wound therapy is to help prevent serious infection postinjury, as well as pathological scar formation to accelerate wound healing. Classic options include medication (i.e., intralesional corticosteroids and intralesional fluorouracil), cryotherapy, surgical excision, and perioperative therapies and laser therapy. Although some of them have proven to be effective, many patients undergoing these treatments suffer from a lot of pain or can be bothered by a high risk of recurrence [94–97]. Thus, developing novel technologies is required. Recent findings on fibroblasts and nanoscale materials may help provide a promising future in scarless wound healing. This strategy largely includes inhibition of fibroblast proliferation, modulation of cell differentiation, and alteration of ECM components.

Generally, fibroblast-related technologies refer to detection and identification of pathological skin repair and wound healing-associated therapy. Regarding pathological diagnosis involving the analysis of mRNA expression, materials include NanoFlares and nucleic-acid-based probe. Through the use of NanoFlares, a type of imaging nanoprobes designed for live-cell detection of mRNA, D.C. Yeo et al. distinguished hypertrophic and keloidal fibroblasts from normal fibroblasts by measuring the expression of connective tissue growth factor (CTGF) [98]. Similarly, Zeng et al. utilized a novel nucleic-acid-based probe in order to achieve this type of distinction. The probe is generally utilized for diagnosis and spontaneous regulation of the abnormal expression (by suppressing the mRNA expression of TGF*β*RI and CTGF) of fibrosis-related mRNA in scar-derived skin fibroblasts [99]. Therefore, these techniques can serve as means of biopsy-free scar diagnosis and eventually help make treatment decisions.

With regard to treatment, fibroblast-related technologies involve skin substitutes, controlled release, and exosomes. With regard to skin substitutes, bioengineered scaffold, hybrid membrane, and marine-derived films are invented. A trilayer PCL-gelatin scaffold mimicking the actual skin structure displayed improved regeneration with an ideal mechanical strength by maintaining a porosity gradient and conducting proper microenvironments [100]. Meanwhile, Li et al. proposed an innovative approach that combines graphene oxide with collagen I and N-acetyl cysteine (NAC), both of which allowed the continuous release of antioxidant NAC. The hybrid membrane exhibits a better antiscar effect, which demonstrates with decreased mRNA expression of profibrotic factors, as well as overexpression of antifibrotic factors [101]. Moreover, application of astaxanthin incorporated collagen film (ACF) and gentamicin incorporated collagen film (GCF) in order promote epithelialization in Wistar rats with full thickness excision and linear incision [102].

The second strategy, controlled release, refers to regulating the same substance across different phases towards opposite effects. This strategy refers to various methods, including multilayered structures, porous design, and photo-induced release. Nanotechniques that play different roles at various stages of wound healing promote regeneration and suppress scarring. A modified formulation of poly (*γ*-glutamic acid), according to electrospun photocrosslinkable hydrogel fibrous scaffolds combined with ginsenoside Rg3 (GS-Rg3), has developed for improved tissue repair function. Reduced scar formation was observed due to sustained release of GS-Rg3, which allows fibroblast proliferation at an early stage but abated angiogenesis and collagen accumulation later [103]. As TGF-*β* signaling pathway participates during whole process, from the activation of transcription factors to fibroblast differentiation and *α*-SMA production, it remains a promising target with regard to scarless wound healing. The exogenous growth factor delivery platform based on coacervate achieves scarless skin regeneration via dual release of TGF-*β*3 and IL-10 at different stages [104]. This type of results is also demonstrated by Zhang et al. using an integrated photocrosslinking strategy. A microcapsule platform is developed with pulsatile release of TGF-*β* inhibitors, demonstrating spatiotemporal specificity across both murine skin wounds and large animal models [105]. Similarly, the controlled release of metformin hydrochloride forms a three-layer scaffold, which alleviates scar formation by downregulating expression of fibrosis-involved genes, including TGF-*β*1, collagen type 1 and 3, fibronectin, and *α*-SMA [106].

Regarding their last strategy, exosomes comprising mRNAs, miRNAs, cytokines, and growth factors are isolated, and their effects on the behavior of fibroblasts are evaluated. The use of exosomes also exerts promising clinical translation [11]. For example, transplantation of exosomes from the human umbilical cord blood plasma (UCB-Exos) accelerates cutaneous wound healing through miR-21-3p-mediated promotion of angiogenesis and fibroblast function [107]. A group of umbilical cord-derived MSCs-derived exosomes demonstrate antiscarring functions via suppression of myofibroblast formation, which may be associated with inhibition of TGF-*β*2/SMAD2 pathway [108].

Other methods that promote scarless wound healing include induction of MSCs-differentiated fibroblast [109], regulation of angiogenesis [110] and TGF-*β*3 expression [111], and M1-M2 phenotype switching of macrophages [112]. Moreover, the silk nanofiber hydrogels loaded with asiaticoside (AC) have been shown to improve efficiency compared to previous liposome systems in reaching scarless wound healing by regulating inflammatory reactions and angiogenesis [113].

## 6. Clinical Trials

Several clinical trials have been carried out or are ongoing that can help clarify the safety, feasibility, and efficacy of fibroblast-based therapeutics in wound healing and skin regeneration. Although clinical guidelines have not included use of fibroblasts, many studies have shown the great potential of fibroblast therapy in clinical applications (Table 1).

A study that enrolled 49 volunteers with circular 5-mm full-thickness wound of unblemished skin underneath both arms who were treated with *α*-CT1 demonstrated dose-dependent decreases in fibroblast movement directionality, which resulted in increased randomness during the migration paths [114]. Meuli et al. recruited seven patients, each with seven wounds. Three wounds were administered fibroblast injection, while the other three wounds used fibroblasts that were seeded on amniotic membrane scaffolds (FAMS). The last one was treated with standard wound care (SWC) (Vaseline gauze). Although increased wound healing was achieved using the first two methods, the fibroblast injection was proven to be superior to FAMS, and a continuous collagen layer was established with better microscopic effects in completely healed wounds [115]. ICX-RHY-013 is an investigational medicinal product that is comprised of viable allogeneic human dermal fibroblast (HDFs) cells that were suspended in HypoThermosol®-FRS. Rubin and colleagues conducted a clinical trial that included eight participants. The participants were divided into two cohorts according to their wound types (cohort 1 with an abdominal incision scar and cohort 2 burn scars with restrictive scar contractures). There were no life-threatening events observed, but there were mild adverse events, including redness and itching. In order to investigate the safety and efficacy of autologous fibroblasts towards severe facial acne scarring, 109 patients were selected and administered with autologous fibroblasts and placebo on either sides of their cheeks, respectively. The autologous fibroblast-treated cheeks earned better scores of Evaluator Live Acne Scarring Assessment (ELASA) and Subject Live Acne Scarring Assessment (SLASA), thereby indicating improved healing conditions with autologous fibroblast treatment.

## 7. Discussion

Skin wound repair is a complex process that can accomplish two major tasks. First, wound repair attenuates skin barrier functions, which effectively protects skin stability and prevents infection. Moreover, wound healing restores the physiological and mechanical properties of skin. Fibroblasts are expected to contract wounds and secrete ECM during the process, but uncontrolled proliferation of fibroblasts and excessive deposition of ECM contributes to the scar formation and should be avoided.

During recent years, numerous studies have been carried out in the field of inhibiting scar formation and have achieved some promising results. Fibroblast heterogeneity, intracellular crosstalk, and signaling pathways have provided some innovative thoughts. However, the exact mechanisms that are involved are still not revealed. Limitations, such as the lack of detection in dynamic change of fibroblast phenotypes and the obscurity of how these lineages are interconnected, remain unsolved. Therefore, further tests during clinical samples are still needed. The treatment of pathological scars remains a thorny and daunting challenge, as most of the current studies, especially clinical trials, have not shown any beneficial effect of treating scarless wound healing. Nevertheless, the recently progressive application of biomaterials has brought some insight into this issue. Special probes are designed as diagnostic tools for pathological scars, and significant therapeutic effects were found in fibroblasts-based technologies concerning skin substitutes, controlled release, and exosomes. Meanwhile, novel techniques and methods, such as lineage tracing, intravital microscopy, single-cell transcription, and epigenetic profiling, can help uncover the underlying mechanisms of skin scarring and provide potential therapeutic targets for regenerative treatment of skin injuries.

The TGF-*β* signaling pathway participates in wound healing, scar formation, and fibroblast reprogramming towards CAFs. While elevated expression of TGF-*β* at the re-epithelialization stage seems to promote wound repair, the continued upregulation at the remodeling phase is related to scarring. While administration of TGF-*β* antibodies during remodeling and the resolution stage can cause significant improvement of skin scarring, treatment at an early stage may cause later cutaneous wound healing [116]. This suggests the importance of the timing of intervention. Meanwhile, TGF-*β* expression is reported to be upregulated in skin cancers such as melanoma. It is worth mentioning that fibroblast sensitivity to TGF-*β* in keloids is higher than normal skin fibroblasts, which causes increased secretion of ECM. On the other hand, melanoma cells appear to be less sensitive to the growth inhibiting effect of TGF-*β*. Therefore, the controlled inhibition of TGF-*β* can be applied clinically as an intervention.

Activated fibroblasts during wound healing, especially scarring and CAFs, share many common cellular features and signaling pathways, but with distinct characteristics. These fibroblasts associated with ECM have a primary role in tissue repair and tumor proliferation. Normal skin fibroblasts can be converted to CAFs under certain condition, with TRAF6, Twist1-Prrx1-TNC loop, and LARP6 acting as inducers, while CLEC2A, SMURF2, and CSL can be used as inhibitors. Therefore, it is likely that controlling proliferation and activities of CAFs may limit tumor progression and improve response to antitumor therapies. In addition, we hypothesize that preventing the transformation of CAFs may reduce progression of tumor at an early stage. Moreover, therapeutic strategies that are aimed at reducing scars may also work in the suppression of cancer. However, a deeper understanding of the main role of fibroblasts in tumors and scars is needed.

## Figures and Tables

**Table 1:** The clinical trials of fibroblast-based therapy in wound healing and scarring.

Conditions	Interventions	Status	Results
Acne scarring of the face	Biological: autologous human fibroblasts (azficel-T)	Completed	Reduced scars in autologous fibroblast cheeks
Restrictive scar contracture Restrictive hypertrophic scar Burn scar contractures Burn scar	ICX-RHY-013	Terminated	Safe
Hypertrophic scarring	AbobotulinumtoxinA 500 UNT	Active, not recruiting	Ongoing
Trophic ulcer Nonhealing wound Nonhealing ulcer of skin	Dermal fibroblasts LED phototherapy	Completed	Ongoing
Burns	Fibroblasts and keratinocytes	Completed	Ongoing
Wound scars	Connexin 43 carboxyl terminal mimetic peptide *α*CT1	Completed	Decreased directionality of fibroblast movement, and the generation of a 3D collagen matrix postwounding that is similar to unwounded skin
Dystrophic epidermolysis bullosa	Fibroblast injection Amniotic membrane scaffolds (FAMS) Vaseline gauze (SWC)	Completed	Establishment of a continuous collagen layer and better microscopic effects

## Data Availability

No data were used to support this study.
